The article "Long duration multi-channel surface electromyographic signals during walking at natural pace: Data acquisition and analysis" was published in 2025. Journal: PLoS One.

# Long duration multi-channel surface electromyographic signals during walking at natural pace: Data acquisition and analysis

**DOI:** 10.1371/journal.pone.0318560

**Published:** 2025-02-12

**Authors:** Francesco Di Nardo, Christian Morbidoni, Grazia Iadarola, Susanna Spinsante, Sandro Fioretti

**Affiliations:** 1 Department of Information Engineering, Università Politecnica delle Marche, Ancona, Italy; 2 Department of Management and Business Administration, Università degli Studi G. d’Annunzio, Pescara, Italy; Opole University of Technology: Politechnika Opolska, POLAND

## Abstract

Variability of myoelectric activity during walking is the result of human capability to adapt to both intrinsic and extrinsic perturbations. The availability of sEMG signals lasting at least some minutes (instead of seconds) is needed to comprehensively analyze the variability of surface electromyographic (sEMG) signals. The current study introduces a dataset of long-lasting sEMG signals recorded during walking sessions of 31 healthy subjects, aged between 20 and 30 years, conducted at the Movement Analysis Lab of Università Politecnica delle Marche, Ancona, Italy. The sEMG signals were captured from ten distinct lower-limb muscles (five per leg), including gastrocnemius lateralis (GL), tibialis anterior (TA), rectus femoris (RF), hamstrings (Ham), and vastus lateralis (VL). Synchronized electrogoniometric and foot-floor-contact signals are also supplied to enable the spatial/temporal analysis of the sEMG signals. The experimental procedure involves subjects walking barefoot on level ground for approximately 5 minutes at their natural speed and pace, following an eight-shaped path featuring linear diagonal segments, curves, accelerations, and decelerations. An advanced analysis of the sEMG signals was performed to test the reliability and usability of the current dataset. The considerable duration of the signals makes this dataset particularly useful for studies where a significant volume of data is crucial, such as machine/deep learning approaches, investigations examining the variability of muscle recruitment during physiological walking, validations of the reliability of novel sEMG-based algorithms, and assembly of reference datasets for pathological condition characterization.

## 1. Introduction

Electromyography (EMG) is acknowledged as one of the main techniques able to supply suitable and reliable biological signals to characterize and study the neuromotor system [1]. Surface electromyography (sEMG) and fine-wire electromyography (fwEMG) could be both employed to identify and describe the recruitment of body muscles during a specific motor task. Nevertheless, fwEMG is quite an invasive and sometimes painful approach. For this reason, it is rarely adopted, except for particular conditions such as capturing the activity of deep muscles or muscles with small cross-sectional areas [2,3]. Specifically, its invasiveness makes fwEMG inappropriate for monitoring dynamic and cyclic tasks, such as walking. On the contrary, sEMG analysis is frequently recommended in this kind of motor tasks because it is non-intrusive, it does not discomfort or hurt patients, it is not difficult to perform, it allows the monitoring of long-lasting tasks, and it permits the recording of muscular activity from a significant proportion of motor-units which is likely representative of whole muscle activity [4–6].

Walking is an activity of huge importance in human everyday life [7]. It is an ordinary movement that involves mainly the lower limb muscles. So, acquiring sEMG signals from those muscles is a prime concern of gait analysis. Indeed, identifying and analyzing muscle activity during gait allows for providing relevant information in clinics, rehabilitation, and recovery from neurological and orthopaedic disorders [8–10]. During physiological walking, myoelectric activity changes considerably from person to person and within the same subject [11,12]. The variability seems to further intensify in pathological conditions [13]. This phenomenon is reported to be the result of the human capability to adapt to both intrinsic and extrinsic challenges and perturbations [14]. The quantification of this wide variability permits to enhance the interpretation of sEMG signals in both physiological and pathological populations. A deeper investigation of sEMG variability could be useful to comprehend the neural basis of muscular synergies [15], to describe the flexibility of musculoskeletal system [16], and to deepen the understanding of processes that the neuro-muscular system adopts to adjust for the ongoing mechanical conditions [17]. The high variability of sEMG signal is one of the main reasons why recent literature is starting to recommend the analysis of muscle recruitment during natural walking lasting at least 3–5 min, not less [18]. Moreover, walking continuously for some minutes allows the subject to move more naturally, as in everyday life. After some strides, subjects start feeling comfortable and walking at their natural pace. Thus, although a few gait cycles might be enough in some applications, the acquisition of EMG signals in more numerous strides is strongly suggested. Despite valuable datasets including sEMG signals being accessible [19–25], to our knowledge free databases composed of long-lasting sEMG signals during walking are not available.

The aim of the present study is to introduce a dataset composed of long-lasting (4-5 minutes) sEMG signals and their analysis. The sEMG signals were recorded during uninterrupted ground walking of 31 young able-bodied subjects in the Movement Analysis Lab of Università Politecnica delle Marche, Ancona, Italy. In addition to the availability of the complete raw sEMG signals from ten different lower-limb muscles (five per leg), the dataset includes synchronized footswitch and knee electrogoniometric signals acquired in the same population, which are useful to achieve a spatial/temporal characterization of muscular recruitment during each walking trial. In a standard protocol of gait analysis, at least four lower-limb muscles are typically considered for sEMG-based evaluations: gastrocnemius lateralis, tibialis anterior, rectus femoris, and hamstrings [18]. The idea is to include one pair of agonist-antagonist muscles for each joint (ankle, knee, and hip). This is possible with only four muscles, since two bi-articular muscles are included in the protocol: rectus femoris (hip and knee) and gastrocnemius lateralis (knee and ankle). Moreover, it is known that vastii muscles have a prominent role in the process of stabilizing patella and knee joint during walking [26]. Thus, the analysis of vastii behavior could add further insight into the comprehension of walking physiology and the etiology of common knee pathologies [27]. For these reasons, sEMG signals from gastrocnemius lateralis, tibialis anterior, rectus femoris, hamstrings, and vastus lateralis are collected and stored in the current dataset.

To test the reliability and the usability of the current dataset, sEMG signal quality was analyzed by evaluating the signal-to-noise ratio (SNR), sEMG frequency content was quantified by the continuous wavelet analysis, and a comparative analysis was performed against the results of acknowledged scientific studies. Further details on the characteristics of the dataset could be found in [28–30].

## 2. Data acquisition

### 2.1. Involved participants

This study is based on gait data recorded from 2011 and 2018 and already used in previous publications. Thirty-one young able-bodied subjects were involved in the study. Detailed anthropometric characteristics of the participants are reported in Table 1. All the participants were students who were used to attending the Movement Analysis Lab. They were selected according to the following inclusion criteria: (i) 20 years old < age <  30 years old; (ii) absence of known locomotor disorders; and (iii) body mass index (BMI) ranging from 18 kg/m^2^ to 25 kg/m^2^ to avoid underweight and overweight conditions. Subjects who communicated manifest disorders, confirmed diseases, pain, or after surgical intervention were excluded.

**Table 1:** Anthropometric information of the participants and task duration.

	Gender	Age (years)	Height (m)	Mass (kg)	Duration (s)	N° of Strides
**Subject 1**	F	25	1.52	45	306	542
**Subject 2**	M	24	1.82	70	317	530
**Subject 3**	F	24	1.58	49	284	455
**Subject 4**	M	24	1.75	76	269	493
**Subject 5**	F	22	1.64	50	320	648
**Subject 6**	F	23	1.63	53	310	546
**Subject 7**	M	27	1.81	66	309	678
**Subject 8**	F	23	1.64	50	254	461
**Subject 9**	M	25	1.81	63	256	608
**Subject 10**	F	24	1.65	60	251	441
**Subject 11**	F	23	1.65	52	260	498
**Subject 12**	F	22	1.66	52	309	613
**Subject 13**	M	26	1.83	76	246	445
**Subject 14**	F	23	1.60	50	313	638
**Subject 15**	F	26	1.70	54	187	398
**Subject 16**	F	23	1.60	50	257	469
**Subject 17**	M	22	1.75	63	311	596
**Subject 18**	F	23	1.68	49	142	256
**Subject 19**	F	26	n.a.	n.a.	188	354
**Subject 20**	F	26	1.68	54	313	606
**Subject 21**	M	22	1.70	66	302	600
**Subject 22**	F	24	1.61	54	122	246
**Subject 23**	M	27	1.74	67	246	432
**Subject 24**	M	29	1.97	86	255	408
**Subject 25**	F	26	n.a.	n.a.	187	383
**Subject 26**	F	24	1.70	60	256	484
**Subject 27**	F	23	1.60	48	246	501
**Subject 28**	M	26	1.83	76	245	445
**Subject 29**	M	21	1.86	86	313	564
**Subject 30**	M	23	1.78	66	246	436
**Subject 31**	F	n.a.	n.a.	n.a.	189	379

n.a. means not available.

Before the experiment, each subject was introduced to the experimental protocol and the motor task to perform and informed of any potential risk. Every subject provided written informed consent. The experiment was performed by trained investigators, using approved and non-invasive protocols. The subject’s welfare was guaranteed during the whole experiment. The data was analyzed anonymously. Authors had no access to information identifying individual participants during or after data collection. Experiments and data acquisition have been conducted according to the ethical principles of the Helsinki Declaration and approved by the local ethical committee.

### 2.2. Test setup

Three different typologies of signals were recorded (Fig 1): basographic, electrogoniometric, and sEMG. The signals were acquired at a sampling rate of 2 kHz and a resolution of 12 bit by the multi-channel recording system Step32 (Version PCI-32 ch2.0.1. DV), Medical Technology, Italy. For the acquisition of the foot-floor-contact signal (i.e., basographic signal), each subject was instrumented with three footswitches (size: 11 × 11 × 0.5 mm; activation force: 3 N, manufacturer: Medical Technology) applied bilaterally beneath the heel (Heel), the first (1^st^ MH) and the fifth (5^th^ MH) metatarsal heads of each foot, as reported in panel A of Fig 2.

**Fig 1:** Schematic representation of the complete acquisition and storage procedure.

**Fig 2:** Acquisition protocol. Footswitches applied bilaterally beneath the heel (Heel), the first (1st MH) and the fifth (5th MH) metatarsal heads of each foot (panel A); Knee electrogoniometer (panel B).

For the acquisition of dynamic knee joint angles in the sagittal plane, an electrogoniometer (accuracy: 0.5°, manufacturer: Medical Technology) was attached to the lateral side of each lower limb (panel B of Fig 2). In some subjects (9 out of 31 subjects, see the.hea file described in the “Data Analysis” section), the hip angle was also measured by applying the same electrogoniometric sensor.

sEMG signals were recorded with single differential probes of fixed geometry constituted by Ag/Ag-Cl disks (manufacturer: Medical Technology, size: 7 × 27 × 19 mm; electrode diameter: 4 mm; inter-electrode distance: 8 mm, gain: 1000, high-pass filter, cut-off frequency: 10 Hz, input impedance >  1.5G Ω, CMRR >  126 dB, input referred noise ≤  1 µ Vrms), and with variable geometry constituted by Ag/Ag-Cl disks (manufacturer: Medical Technology, minimum inter-electrode distance: 12 mm, gain: 1000, high-pass filter, cut-off frequency: 10 Hz, input impedance >  1.5G Ω, CMRR >  126 dB, input referred noise ≤  200 nVrms). sEMG signals were further amplified and low pass filtered (cut-off frequency 450 Hz) by the recording system. Probes with fixed geometry were applied over gastrocnemius lateralis (GL), tibialis anterior (TA), and Hamstrings (Ham) whereas probes with variable geometry were applied over rectus femoris (RF) and vastus lateralis (VL), as depicted in Fig 3. It is worth specifying that the sEMG signal indicated with “Hamstrings” reflects the global combined function of the hamstrings muscle group during walking, including the medial (semimembranosus and semitendinosus) and lateral (biceps femoris) muscles, rather than isolating the sEMG signals from individual muscles within the hamstring complex.

**Fig 3:** sEMG acquisition protocol. sEMG probes with fixed geometry were applied over tibialis anterior (TA), gastrocnemius lateralis (GL), and Hamstrings (Ham) and probes with variable geometry were applied over rectus femoris (RF) and vastus lateralis (VL).

Before positioning the probes, the skin was shaved, cleaned with abrasive paste, and then wet with a soaked cloth. To ensure proper electrode-skin contact, electrodes were dressed in highly conductive gel. Electrode location and orientation over the muscle with respect to tendons, motor point, and fiber direction were accomplished to the European Recommendations for Surface ElectroMyoGraphy (SENIAM) [31]. Footswitches and electrogoniometers were positioned following the standard procedure indicated by the manufacturer of the system. All these sensors and signals converge into the Patient Unit of the multi-channel recording system. This Patient Unit (Fig 1) is positioned at the lower back, anatomically corresponding to the lumbar spine. This placement situates the device just above the sacral region and superior to the gluteal muscles, ensuring a strategic alignment that follows the natural curve of the lumbar region. The Unit is secured with an adjustable elastic belt that wraps around the subject’s waist. This belt ensures a stable fit, allows for slight adjustments to accommodate various body types and maintains comfort, while minimizing the side-to-side and up-and-down movement of the Unit during physical activities, especially while walking.

Signals were checked for quality and sensor positioning and regulated as necessary. sEMG probes, footswitches, and electrogoniometers are parts of the same acquisition system (Step32 - Version PCI-32 ch2.0.1. DV, Medical Technology, Italy); thus, all the signals are acquired synchronously. The sampling rate of 2 kHz allows to describe the full bandwidth of the sEMG signal.

To mitigate cross-talk, electrode placement followed SENIAM guidelines [31], prioritizing electrode orientation and muscle alignment. Moreover, the procedure indicated in [32] was also adopted. Once the EMG probes had been positioned, crosstalk verification was conducted through visual examination. Cross-talk was presumed if simultaneous activity with similar amplitude variations was observed in two muscles within the same limb section. In this case, double differential probes were employed to enhance spatial selectivity, and the signal obtained from these probes was compared against that of the single differential ones. Confirmation of cross-talk was established when the double differential signal displayed a noticeably reduced amplitude; in such cases, the signal was disregarded.

### 2.3. Acquisition protocol

Before starting a trial, subjects were asked to stand in their comfortable posture for 5 seconds. Then, volunteers were encouraged to walk barefoot uninterruptedly on level ground for around 5 minutes. The average trial duration (± standard deviation, SD) over the whole 31-subject population is 258 (± 53) s. Details of the trial duration are reported in Table 1. One single trial was performed by each subject. Subjects were given no specific indication about speed, pace, acceleration, deceleration, or reversing. They were only asked to follow freely an eight-shaped path like the one described by the black feet in Fig 4. No markers or signs on the floor were added. The shape of this path (including acceleration, deceleration, and reversing) and the long duration of the trial were chosen to allow the subject to move more naturally, as in everyday living. Despite subjects being given no indication, three different paces adopted by the subjects were observed during the experimental trials. The three zones characterized by the three different paces are superimposed to the eight-shaped path in Fig 4 to help the comprehension of pace variability during this walking task: the red zones, where subjects were used to curving or reversing; the yellow zones, where subjects were used to accelerating and decelerating; and the orange zone, where subjects were used to walk following linear diagonal segments. The eight-shaped path was indeed intentional to introduce variability in sEMG patterns and emulate everyday walking with natural deviations.

**Fig 4:** The walking path adopted during the experimental trial. Orange indicates the zone where subjects walked following linear diagonal segments; yellow indicates the zones where subjects accelerated or decelerated; and red indicates the zones where subjects curved or reversed.

## 3. Data analysis

The dataset is composed of raw walking signals recorded from 31 young healthy subjects. Following the PhysioNet requirements [29], the files are provided in waveform database (WFDB) format. Specifically, two WFDB files are provided for each subject, with “.dat” and “.hea” extensions. For example, for the first subject (S1), the two files S1.dat and S1.hea are available. The.dat file is structured as a data matrix composed of 14 rows. Each row includes a whole signal (basographic, electrogoniometric, or sEMG) according to what is reported in the correspondent.hea file. The.hea file provides the sampling rate (in Hz) and the number of samples for each signal and then describes the order in which the signals are stored (from row 1 down to row 14). sEMG signals are expressed in μV; foot-switch signals are expressed in V; and electrogoniometric signals are expressed in degrees. Footswitch and electrogoniometric data are provided to allow users to achieve a spatial/temporal characterization of muscular recruitment during walking. Footswitch, electrogoniometric, and sEMG signals are synchronized. The basographic signals from footswitches were converted to four levels and processed to segment and classify the different gait cycles under the acknowledged procedure introduced in [33]. Briefly, the procedure is based on the computation of the least significant bit (LSB), defined as the difference between the maximum and minimum values of the basographic signal (expressed in V), normalized by the number of quantization levels provided by the footswitches, which in this case is 8 (2 values, ON or OFF, for each of the three footswitches leading to 2^3 =  8). This allows for the extraction of 8 gait phases from the =basographic signal recorded by the footswitches. Then, an additional quantization process was performed, by grouping some of these 8 levels in order to achieve 4 phases. Each new level corresponds to a specific phase of the foot-floor contact: Heel contact (H), Flat foot contact (F), Push off (P), Swing (S). The complete and detailed procedure is reported in [33]. The total uncompressed size of the whole dataset is 427.0 MB. A text file with the anthropometric information of the participants reported in Table 1 is also included. An example of each typology of signal visualized in a single stride of a representative subject (subject 12) is shown in Fig 5.

**Fig 5:** An example of recorded signals included in the proposed dataset: basographic (panel A), electrogoniometric (panel B), and sEMG (panel C) signals.

### 3.1. SNR analysis

sEMG signal quality was tested by evaluating the signal-to-noise ratio (SNR). The SNR of each raw signal was computed (in dB) using the approach described by Bonato et al. [34], which quantifies it as the logarithm of the ratio between the square of the standard deviation (SD) of the sEMG signal and the square of the SD of the noise:


$$SNR=10*\log\frac{\left({\text{σ}}_{signal}^{2}\right)}{\left(\sigma_{noise}^{2}\right)}$$ (1)

where ${\text{σ}}_{noise}$is the SD of the noise and ${\text{σ}}_{signal}$is the SD of the actual signal. In this current study, this method was applied exactly as described, without any additional filtering of the signal (aside from the hardware filtering described in section 2.2) or outlier removal. The only contribution made by the authors was in selecting which part of the signal to use for calculating the SD of the noise and which part for calculating the SD of the signal, as follows. Before the beginning of the experimental trial, subjects were asked to stand in their comfortable posture for 5 seconds (i.e., around 10000 samples). These 10000 samples were considered as noise. Then, the first 10000 samples of the sEMG signal were visually inspected to identify potential undesired muscle activations or spikes. ${\text{σ}}_{noise}$was computed in this segment of 10000 samples, excluding undesired muscular activations and spikes. ${\text{σ}}_{signal}$is computed in the remaining samples of the signal from 10000 to the end. SNR value computed in each signal is reported in Table 2.

**Table 2:** SNR values for all sEMG signals.

Signal to noise ratio - SNR (dB)												
Subject	TAleft	GLleft	RFleft	Hamleft	VLleft	TAright	GLright	RFright	Hamright	VLright	Mean	SD
**1**	22.6	12.4	5.9	11.5	25.0	28.4	11.4	12.5	12.8	22.8	16.5	7.5
**2**	22.1	14.2	11.6	10.4	13.4	21.7	23.2	16.2	16.7	19.1	16.9	4.5
**3**	21.7	14.0	16.3	13.9	22.6	22.1	9.9	19.9	31.2	23.5	19.5	6.1
**4**	23.4	12.1	14.4	9.1	21.0	25.6	12.7	14.6	9.2	17.8	16.0	5.8
**5**	19.7	13.7	14.2	10.5	22.0	14.6	10.6	12.4	8.0	15.5	14.1	4.2
**6**	22.9	20.9	15.7	16.8	24.8	10.3	26.3	13.7	12.6	23.5	18.8	5.6
**7**	23.6	19.9	12.1	15.9	18.6	21.4	17.7	9.7	14.4	18.1	17.1	4.2
**8**	20.2	16.9	21.2	13.8	32.0	24.1	12.1	18.6	16.3	17.0	19.2	5.7
**9**	32.7	16.0	8.9	10.6	25.8	26.7	17.0	24.7	10.4	21.0	19.4	8.1
**10**	25.8	10.6	19.4	9.0	23.7	25.5	14.9	15.0	7.6	13.8	16.5	6.8
**11**	20.5	15.7	17.1	10.4	13.7	22.3	12.4	9.8	11.8	11.9	14.6	4.2
**12**	24.9	10.5	18.7	12.4	25.3	23.9	10.8	19.0	8.4	22.8	17.7	6.6
**13**	24.0	21.8	22.6	6.3	22.5	26.6	20.1	14.5	8.0	23.7	19.0	7.0
**14**	25.0	19.4	15.8	16.2	24.1	23.4	15.2	14.5	16.7	15.9	18.6	4.0
**15**	26.7	19.6	20.2	18.1	31.2	24.7	18.4	11.3	12.8	20.9	20.4	6.0
**16**	22.5	17.3	19.5	12.0	14.3	23.3	16.7	22.8	14.2	10.2	17.3	4.7
**17**	27.2	12.0	15.3	10.9	25.0	26.0	11.7	12.3	10.7	15.2	16.6	6.7
**18**	25.8	20.4	17.8	12.0	27.7	25.6	22.6	15.1	19.9	19.7	20.7	4.9
**19**	28.3	22.3	24.3	18.3	25.6	26.9	23.1	19.2	17.9	20.6	22.6	3.6
**20**	13.5	9.1	6.9	3.3	14.8	5.3	9.0	2.9	2.1	9.7	7.7	4.4
**21**	23.8	16.2	14.3	11.9	20.8	26.5	16.4	9.0	13.0	15.5	16.7	5.5
**22**	24.2	27.3	20.8	11.4	24.3	24.7	25.4	20.2	11.4	27.7	21.7	5.9
**23**	22.7	17.5	17.3	5.4	29.7	27.9	18.3	5.4	4.1	20.1	16.9	9.2
**24**	24.2	15.9	11.3	7.8	10.0	24.4	12.3	7.7	10.7	9.5	13.4	6.2
**25**	19.2	15.9	22.1	7.0	25.0	24.7	19.4	16.6	25.6	25.5	20.1	5.9
**26**	28.5	11.4	14.7	10.5	20.5	32.7	21.4	12.3	8.1	16.2	17.6	8.1
**27**	25.8	14.5	27.0	13.4	28.4	24.1	18.5	28.4	12.7	22.4	21.5	6.3
**28**	24.0	21.8	22.6	7.1	22.5	26.6	20.1	14.5	7.7	23.7	19.1	6.9
**29**	23.8	15.6	15.9	14.8	17.7	21.2	9.6	12.0	11.3	21.8	16.4	4.7
**30**	28.1	14.7	18.9	11.8	12.2	25.1	10.9	14.7	9.4	20.0	16.6	6.3
**31**	20.2	13.1	12.3	7.5	12.1	23.5	14.1	19.2	11.2	24.0	15.7	5.6
**Mean**	23.8	16.2	16.6	11.3	21.8	23.5	16.2	14.8	12.5	19.0		
**SD**	3.5	4.2	4.9	3.7	5.9	5.2	5.0	5.4	5.8	4.8		

Mean SD is computed for each muscle over all subjects and for each subject over all muscles.

A common guideline indicates that SNR higher than 10 dB could be considered suitable for most clinical and research applications of sEMG signals. This SNR value indicates that the signal amplitude is at least 10 times higher than the background noise, providing a relatively clear distinction between the desired muscle activity and the unwanted noise components. However, lower SNR values, such as 5–10 dB, may also be considered adequate in specific experimental conditions. The last two rows in Table 2 show that the average SNR value over the whole population is higher than 11 dB for each muscle. Moreover, only 10% of SNRs in Table 2 are lower than 10 dB and a negligible percentage of SNRs (0.97%) is lower than 5 dB.

### 3.2. Frequency analysis

The acquired sEMG signals were validated also using the quantification of their frequency content. First, the basographic signals were processed to segment and identify the different gait cycles following the acknowledged procedure introduced in [33]. For each muscle and each gait cycle, the time-frequency energy density of the signal was identified through the scalogram function provided by the continuous wavelet analysis [35]. Moreover, the maximum energy density was assessed, as the time-frequency interval in which the energy density exceeds 75% of its peak value over the gait cycle. An example of a wavelet scalogram for two muscles representative of distal-leg muscles (tibialis anterior) and proximal-leg muscles (rectus femoris) in a random stride is depicted in Fig 6.

**Fig 6:** Example of time-frequency representation of sEMG signal. Energy density of the sEMG signal is represented through wavelet scalogram in a random stride for two representative muscles. Gait cycle percentage and frequency content are reported in the horizontal plane. Normalized color-level coded scale represents the amplitude of energy density; red =  maximum energy density; blue =  minimum energy density.

For all muscles and all strides, the energy density of sEMG signal is completely included in the range [0–500] Hz, which is the typical frequency content of this electrophysiological signal [33]. Specifically, the maximum frequency detected in a single stride ranges from around 150 Hz up to almost 500 Hz, in line with what was reported in [35]. The maximum energy density ranges in [60–170] Hz for GL, [60–220] Hz for TA, [65–220] Hz for RF, [60–185] Hz for Ham, and [65–220] Hz for VL.

Despite the frequency content changing from muscle to muscle, a common frequency band of [65–170] Hz could be identified among all muscles, consistent with EMG literature [36,37]. Possible motion artifacts typically reported in low frequency ([0–15] Hz), ECG interference (typical in trunk muscles but very rare in leg muscles, [0–30] Hz), and power line noise (50 Hz) are not perceivable in these signals.

### 3.3. Comparison to other datasets

To test the reliability of the current dataset, a comparative analysis was performed against the results of acknowledged scientific studies with walking conditions as similar as possible to the ones considered here. In those studies, muscle activation intervals are typically expressed as a function of the gait cycle. Thus, the basographic signals were processed to segment and classify the different gait cycles under the acknowledged procedure introduced in [33]. Furthermore, for each gait cycle the main four gait phases were chronologically identified: Heel contact (H), Flat foot contact (F), Push off (P), and Swing (S). Electrogoniometric signals were low-pass filtered (FIR filter, 100 taps, cut-off frequency of 15 Hz). Most of the gait studies reported in literature were performed during straight walking. For a suitable comparison with those studies, it was necessary to detect and discard non-straight or altered cycles from the present dataset, like those relative to deceleration, acceleration, and reversing. A multivariate statistical filter [33,38] was adopted to test knee angles and gait phase durations from every stride of the subject’s walking, by comparing them with the mean value computed on each single subject. If knee angles and/or gait phases in the single stride were significantly different from the mean value, that stride was rejected. sEMG signal was high-pass filtered (FIR filter, 100 taps, cut-off frequency of 20 Hz) to reduce movement artifacts. Muscle activation intervals were computed in each gait cycle by the application of a widely adopted double-threshold statistical detector to sEMG signals [34]. Onset and offset instants of activation were expressed in percentage of gait cycle. Then, mean activation intervals over all the strides of the population were computed as follows: (i) since the number of muscle activations is cycle (stride) dependent [38], for each subject gait cycles are grouped by the number of activation intervals; (ii) for each subject, onset and offset instants of each activation were averaged over each group; (iii) values computed in (ii) were averaged over the whole population of 31 subjects, respecting the grouping criteria; (iv) standard error was computed; and (v) mean data for each group were plotted as a function of gait cycle percentage. This approach to data organization is known as Statistical gait analysis (SGA). Results are depicted in the following Figs 7 and 8.

**Fig 7:** Activations of proximal-leg muscles. Average (± standard error) activation intervals for the three main modalities of activations for rectus femoris (upper panel), hamstrings (middle panel), and vastus lateralis (lower panel) during gait cycle.

**Fig 8:** Activations of distal-leg muscles. Average (± standard error) activation intervals for the three main modalities of activations for gastrocnemius lateralis (upper panel) and tibialis anterior (lower panel) during gait cycle.

Overall, the activation intervals follow the typical pattern reported for these five muscles by acknowledged physiological references in the literature [3,4]. Despite this first confirmation, a more reliable comparison should be made against more recent results proposed in the literature with the same approach (SGA), but with different datasets. Figs 7 and 8 clearly illustrate how the same muscle can exhibit different activation patterns (and thus sEMG signal with different characteristics) across various strides. Specifically, this analysis shows distinct modalities of activation, characterized by one, two, or even three activation intervals per gait cycle in different strides for the same muscle. This variability underscores the complexity of muscle recruitment during natural walking and provides empirical evidence of the non-uniformity of sEMG signals. Only the extended duration of data acquisition allowed to perform the SGA, enabling it to identify and categorize multiple activation modalities per muscle with statistical reliability. To be useful, SGA requires the acquisition of sEMG signals in numerous strides. Thus, all SGA-based studies are typically performed on datasets consisting of long-lasting sEMG signals. This allows for a more suitable comparison with the proposed dataset, also composed of long-lasting sEMG signal. Unfortunately, despite detailed research on the web, we were not able to find free downloadable datasets for direct comparison. Different sEMG datasets during walking are available. However, they are limited by short duration of the trials (only few consecutive strides per subject), and/or small number of muscles considered, and/or by considering treadmill walking [19–25]. The current comparison was performed against the results of acknowledged SGA-based studies [32,39–41] and reported in Table 3, in terms of onset and offset of each activation interval of the two most frequent activation modalities for each muscle.

**Table 3:** Validation versus SGA-based studies.

	Current study	Agostini et al. 2010 [32]	Di Nardo et al. 2013 [40]	Strazza et al. 2017 [41]
**GL1**	12.1-47.2	–	11.2-47.8	–
**GL2**	7.5-34.0; 66.7-79.2	7.3-37.1; 66.9-80.0	6.5-36.3; 68.3-80.7	–
**TA2**	2.6-16.1; 61.4-98.1	0-15.2; 60.5-100	1.69-11.0; 58.6-98.8	–
**TA3**	0.9-7.2; 43.8-59.9; 74.1-100	0-9.3; 48.8-65.3; 79.0-100	0.5-7.4; 41.9-57.1; 72.6-99.9	–
**RF2**	0.9-20.0; 79.7-99.1	**–**	**–**	1.9-24.2; 80.2-98.0
**RF3**	0.2-17.0; 45.0-58.7; 85.0-99.5	0-17.9; 46.4-59.2; 85.1-100	–	0-15.9; 44.8-57.3; 85.6-99.6
**Ham2**	3.7-25.2; 80.8-98.3	0-27.4; 77.5-100	–	7.3-18.2; 76.9-98.0
**Ham3**	0-17.0; 32.8-44.4; 82.2-99.4	0-16.7; 35.5-47.9; 79.6-100	–	1.9-8.3; 41.7-53.2; 79.0-99.4
**VL2**	0-18.7; 82.8-100	0-19.6; 83.7-100^*^	–	0-20.1; 81.5-100
**VL3**	0-15.2; 35.1-47.6; 83.5-100	**–**	–	0-17.6; 38.9-43.1; 81.8-100

The first column reports the name of the considered muscle associated to a number which represents the number of activation intervals (for example, GL1 means activation intervals of gastrocnemius lateralis with only 1 activation in the gait cycle). In each cell of the table, onset and offset of the activation intervals (separated with a hyphen) are reported in order of appearance in the gait cycle.

* Agostini et al. analyzed vastus medialis in place of VL. All the data in the table are expressed as % of gait cycle.

The third column in Table 3 reports the results of the EMG-based study performed by Agostini et al. [32] in a population of 100 healthy school-age children. The acquisition was accomplished with the same model of the recording system used in the current study (Step32, Medical Technology); the experimental procedure and sEMG analysis (SGA) were also the same. Trial duration was 2.5 minutes. The only actual difference between the two datasets is the age of the subjects (mean ±  SD): (24.2 ±  1.9) years in the current study, versus (9.0 ±  1.4) years in [32]. However, many studies indicated that the mature pattern of muscle activity is usually achieved around six years in normally developing children [32,42–44]. Thus, given the difficulty encountered in finding suitable signals for comparison, this rich dataset could be considered as a reliable reference. Results in Table 3 (column 2 versus column 3) show that the assessment of activation intervals provided by the two studies is substantially superimposable for each muscle, strengthening the quality of the proposed dataset. A further SGA-based study could be useful to evaluate the quality of the current dataset [39]. This other study includes a population of 18 young healthy subjects (10 females and 8 males, age range 20-30 years, trial duration =  3 minutes) which matches the sample considered here. Nevertheless, the manuscript presents the result only in graphical forms (figures) and it is not feasible to extract the detailed onset and offset instants of activation to compare with. However, the comparison performed by visual inspection indicates a total agreement between the results of the present analysis and the one reported in [39]. To be thorough, the results of two previous SGA-based studies [40,41] of the same group of researchers of the current study have also been reported in Columns 4 and 5 of Table 3. The first study [40] focuses on the analysis of ankle muscles during ground walking. Fourteen healthy volunteers were included (mean age ±  SD): (23.9 ±  2.3) years; male-female ratio: 7/7, task duration: 5 minutes. Strazza et al. [41] consider a population of 30 healthy subjects (15 females and 15 males, age range 20–30 years, trial duration =  5 minutes). As highlighted in Table 3, these results further support the reliability of the current dataset. However, comparison results could be influenced by the fact that part of these signals have been included in the current dataset.

To conclude this section, it is worth mentioning that signals from the current dataset were already used in numerous published studies on human walking, including the statistical evaluation of ankle muscle activation intervals [40], the quantification of muscle co-contraction [41], and as a control group for examining the variability of muscular recruitment in hemiplegic walking [13]. In more recent studies, these signals were employed as input to neural networks to classify and predict gait phases from sEMG signals [30,45], as well as to evaluate the reliability of novel algorithms for muscular activation detection [35].

## 4. Data usage notes and data limitations

The substantial duration of these signals renders this dataset highly suitable for Compressed Sensing [46], or Machine Learning approaches that rely on extensive data volume. Additionally, the dataset can be utilized to serve as a reference dataset for characterizing pathological conditions as well as to analyze and quantify the variability of muscle recruitment during normal walking. Specifically, methods like Lyapunov exponent (LyE), approximate entropy (ApEN), and detrended fluctuation analysis (DFA) are powerful tools for assessing signal variability and complexity. Given that the present dataset is publicly available through PhysioNet, it could be possible to compute these non-linear figures on the dataset to analyze variability and complexity.

Despite the care employed in the experimental procedure, it is necessary to report some limitations noticed in the current dataset. The first issue concerns the population, which is not perfectly gender-balanced (19 F vs. 12 M). Differences in muscle activity and gait patterns between genders are well-documented, and this could potentially influence the generalizability of sEMG-based findings. However, we would like to emphasize that the primary objective of this work is to introduce a free-available dataset, showcasing its complexity, uniqueness, and potential applications, rather than to provide clinical or research indication or results (which could be interesting for future studies but currently go beyond the scope of the present work). The analyses conducted here were intended solely to highlight the dataset value and its capacity to support further studies. Notably, this dataset could also facilitate future research focused on gender-specific muscle recruitment during walking, as it allows for balanced subgroup analyses (e.g., 12 females vs. 12 males), as done in previous works by this same research group [47].

Then, participants were not given specific instructions regarding their walking speed, pace, or acceleration. The lack of standardized instructions may introduce variability in gait patterns among participants, affecting data consistency. However, the primary objective of this study was to create an sEMG dataset that captures muscle activity while walking as naturally as possible, closely reflecting the gait patterns adopted in daily life. The variability due to the lack of standardized instructions is therefore not seen as a limitation but rather as an inherent strength of the dataset. By including a broader range of walking behaviors, the dataset provides a richer and more realistic foundation for research that aims to understand muscle recruitment in real-world scenarios. Nonetheless, it is important to remember that the analyses conducted here to highlight the potential of the dataset could be influenced by the variability of gait patterns. Therefore, potential users of this dataset should be aware of its context and apply it appropriately in their studies.

In the current study, a wired multi-channel recording system was used to capture sEMG signals, electrogoniometric data, and foot-floor contact signals. It is recognized that the presence of wires can theoretically introduce constraints or affect gait to some extent. Thus, careful attention was given to the management of the cables in order to minimize any impact on the participants’ natural gait. Specifically, the cables were secured and organized to reduce tension and allow freedom of movement. They were routed along the body and affixed in such a way as to prevent excessive slack or interference with the participants’ stride. This approach was intended to ensure that the walking experience remained as natural as possible. It is worth also mentioning that the extended duration of our sEMG recordings helps mitigating initial sensor-induced discomfort, allowing participants to achieve more natural gait patterns over time. At the end of the test, indeed, no significant restrictions were reported by the participants during the trials.

The last two columns in Table 2 show that the average SNR value over all muscles is higher than 13 dB for each subject. Only for subject 20, mean SNR is lower than 10 dB (7.7 dB) and some sEMG signals are characterized by a very low SNR value ( < 5 dB, left Ham, right Ham, and right RF). The use of these signals is recommended only after selective noise filtering has been applied.

Saturation of sEMG signal was identified on two occasions: in the left GL of subject 2 from sample 187280 to sample 248245 and in the right Ham of subject 3 from sample 23343 to sample 88880. However, the cases of signal saturation involve only two sEMG signals out of a total of 310 recorded sEMG signals across the entire dataset. Therefore, we believe that these isolated instances do not compromise the overall quality and reliability of the dataset. Moreover, in the left Ham of subject 16, a high spike probably due to an unexpected interference is identified at sample 260730, lasting around 300 samples. However, it should be noted that this interference lasts for only 300 samples. We consider this spike negligible compared to the total signal duration of approximately 514000 samples, given its minimal impact on data integrity. The presence of these signal issues advises caution when using specific portions of the data, recommending data-cleaning techniques and selective exclusion of compromised segments.

Subject 18 interrupted her walking trial at around sample 240700 due to the detachment of one of the sensors. Therefore, data from that sample onwards are no longer reliable. Some of right (around sample 165363) and left (around sample 176765) footswitches detached due to excessive sweating of the subject 22. Thus, from these samples onwards, the basographic signal is reliable only for discriminating the two main phases of the gait (stance and swing) and not for a more detailed description. No further significant issues were detected. Users are advised to consider all these issues when utilizing the current dataset.

## 5. Code availability

The basic algorithm code developed for identification of each stride from the whole basographic signal is available at the general-purpose open repository figshare [48]. The main purpose of the algorithm is to extract, from the basographic signal, the starting sample of each stride (and also the end sample, since the strides are consecutive.) in order to segment the sEMG signal in strides. The script runs in Matlab environment with a minimal interactive interface. At the first level, the user is asked to enter the number of the stride to analyze. Then, the user is prompted to indicate the channel number (i.e., the row of the matrix) of the basographic signal to display (right or left according to the protocol reported in the.hea file) and the corresponding channel for the muscle. Finally, the user needs to enter the name of the input.mat file. At the end of the procedure, the starting sample of each stride is saved in the variable “indice” and a figure for visualizing the basographic signal and its corresponding sEMG signal in the selected stride is provided.
